# Research on Application Experience Design of Ice and Snow Sports Equipment Based on Bee Colony Model

This article has been retracted.

**DOI:** 10.1155/2022/8760053

**Published:** 2022-07-20

**Authors:** Yuanjing Li, Jintian Yang, Shanshan Gao

**Affiliations:** ^1^The Department of Physical Education, Hebei University of Economics and Business Shijiazhuang, Shijiazhuang 050061, China; ^2^Guangdong Technology College, Zhaoqing 526100, China

## Abstract

Sports equipment is the key to the smooth development of ice and snow sports. With the rapid development of social economy and the improvement of people's living standards, the demand for ice and snow sports equipment is increasing day by day. This article presents an improved method based on the chaos theory and the bee colony algorithm to quantify the application experience design of ice and snow sports equipment and reduce the influence of uncertain factors on the design results. First, the chaos theory can establish the dataset of application experience design and analyze the discreteness of the set. According to the bee colony algorithm, the dataset is divided into several groups, and each group obtains the best application experience design by using the design optimization strategy. Finally, the results are mixed to obtain the final experience design results. Through MATLAB simulation analysis and verification, the improved bee colony model can improve the accuracy of application experience design of ice and snow sports equipment in an uncertain environment, shorten the overall design time, and meet the requirements of application experience design of different ice and snow sports equipment. Therefore, the model proposed in this paper is suitable for the application experience design of ice and snow sports equipment.

## 1. Introduction

With the improvement of living standards, the demand for ice and snow sports equipment is increasing day by day, and it is developing in the direction of intelligence and complexity, so it is particularly important to judge the application experience design of ice and snow sports equipment. The key to the application experience design of ice and snow sports equipment is to judge the experience degree and the type of ice and snow sports equipment [1]. The logistics chaos theory can not only judge the nonlinear relationship between the application and application design of ice and snow sports equipment, but also experience the nonlinear and complex problems of design. It is the main method to judge the application experience design of ice and snow sports equipment at present. Literature research shows that the chaos theory of logistics can classify the application experience design of ice and snow sports equipment, shorten the design time, and improve the overall effect of experience design. However, the complexity of subjective factors and uncertain factors will affect the selection of model parameters, and then affect the final judgment results of ice and snow sports equipment in the process of classification of ice and snow sports equipment application experience design by the logistics chaos theory. Some scholars also put forward the artificial bee colony algorithm. Although this algorithm can judge the application experience design of ice and snow sports equipment, the judgment ability of this method is greatly reduced under uncertain and complex conditions [2]. Therefore, some scholars put forward an improved strategy of the bee colony algorithm to improve the judgment effect of artificial bee colony algorithm. Some scholars put forward the chaos theory of logistics, which is integrated with the bee colony algorithm [3] to experience the uncertainty and complexity of design and improve the reliability of design. Based on this, this paper tries to integrate the bee colony model with the logistics chaos theory to comprehensively judge the application experience design of complex ice and snow sports equipment, and the results are shown in Table 1.

From the above analysis, we can see that the bee colony algorithm has become the main method in the research of ice and snow sports design, and its application depth is increasing day by day. The application of the bee colony algorithm in ice and snow sports equipment can realize continuous analysis and preprocess massive data to get more accurate results. However, there are unrelated unstructured data in massive data, which will affect the accuracy of analysis results and restrict the implementation of the bee colony algorithm. In order to solve the above problems, this paper combines the chaos theory with it, eliminates irrelevant data, and improves the processing effect of previous data. At present, there are many research methods of ice and snow sports equipment application experience design, such as statistical methods, survey methods, and video methods. However, the above methods are qualitative methods and lack of comprehensive analysis, so it is impossible to accurately judge the results. In order to solve the above problems, this paper integrates the bee colony algorithm and the chaos theory into the application experience design of ice and snow sports equipment, aiming at improving the accuracy of the results.

## 2. Related Concepts

### 2.1. Bee Colony Theory

Logistics chaos theory is a comprehensive improved theory put forward in the 1990s, which can comprehensively analyze experience design samples and is suitable for complex data type analysis [4]. In the early 1990s, the logistic chaos theory was widely used in the fields of machinery, electronics, computing, communication, and so on. The logistic chaos theory can accurately calculate the relationship between data, judge the logicality between data structures, and improve the accuracy of calculation results. Simply put, the bee colony theory is an intelligent algorithm, which belongs to the research content of bionics field. Because the bee colony algorithm has the characteristics of randomness and discreteness, the final result is more accurate, and it is suitable for dividing massive data and persistent data. At present, the bee colony theory has been applied in the fields of machinery, computer, aerospace, and so on and achieved satisfactory results. The bee colony theory mainly imitates the process of bee seeking honey source and analyzes the behavior of bees. Bees are divided into leading bees, collecting bees, and telling bees. In the process of changing roles of bees, chaotic analysis should be carried out on the results of honey sources, so as to expand the scope of honey collection. Therefore, the results of the bee colony theory and the chaos theory can not only improve the accuracy of the results, but also expand the search range and improve the comprehensiveness of the results. The bee colony theory belongs to the intelligent algorithm, and the chaos theory belongs to the data processing method, which complement each other and can mine data information more deeply and improve the accuracy of the results.

**Theorem 1 .**

Assuming experience design samples i is any natural number, arbitrary sample data $d_{i}\in \overset{⟶}{R}$, the ultimate expectation of experience design *Q*_*i*_ ∈ [−1,1], and the influencing factors of experience design samples *b*_*i*_ ∈ [1, +*∞*]. Ice and snow sports equipment *K*(*x*_*i*_) will change space under different influencing factors *L*(*x*_*i*_) , and calculate the best effect of experience design to maximize its value *S*_*f*_ [5]. The specific calculation formula is given as

(1) $$\begin{array}{c} S_{f}=w\cdot f\left(x_{i}\right)+\lambda , \end{array}$$

where *w* is the weight of the experience design and *λ* is the threshold of experience design. At that time |*S*_*f*_|=1, the design effect of experience design samples was the best, and the classification interval of experience design samples was the largest [6].

**Theorem 2 .**

If the design requires that the adjustment coefficients *ξ*_*i*_ are evenly distributed in the range of [0,1], it means that the experience design samples are correctly classified, while those distributed in are incorrectly classified [1, +*∞*], and the best effect of experience design *S*_*f*_ can be expressed as

(2) $$\begin{array}{c} \left\{\begin{array}{c} ∴\max S_{f}=w\cdot K\left(x_{i}\right)+\lambda \sum \xi_{i},\\ ∵w\cdot K\left(x_{i}\right)\in \left[0,1\right], \end{array}\right. \end{array}$$

where C is the bad evaluation factor of sports, which mainly regulates the relationship between the misclassification rate of experience design samples and influencing factors.

**Theorem 3 .**

If ice and snow sports equipment satisfies the Mercer condition, then the linear space *L*(*x*_*i*_) of influencing factors can be expressed as

(3) $$\begin{array}{c} \left\{\begin{array}{c} \max L\left(a\right)=\sum a_{i}-\sum a_{ij}q_{ij}K\left(x_{i}\right),\\ ∴a_{i}=z_{i},a_{i}\in \left[0,+\infty \right], \end{array}\right. \end{array}$$

where *L*(*a*) represents the angle of original data points and experience design points, the parameter C in the logistics chaos theory is the key to the application experience design of ice and snow sports equipment, and it is also the main parameter optimized in this article.

### 2.2. Improved Bee Colony Model

The artificial bee colony algorithm mainly analyzes the key indicators, including ergonomic analysis, sports equipment function, sports equipment materials, equipment safety, equipment price, and equipment appearance. During initialization, the number of sports equipment and experience design is the same [7], and different sports equipment intelligently obtains an optimal experience design. First of all, randomly generate sports equipment, design experience design near sports equipment with better satisfaction value, and eliminate “poor” design schemes through competition, about 1/2 of the number. Then, the sports equipment function adopts the strategy of roulette to choose the best experience design, gives the corresponding weight, and carries out greedy design around it to produce 1/2 experience design [8]. Finally, give up the experience design of sports equipment that does not meet the threshold, and design sports equipment in other directions.

Assuming that the initial number of sports equipment and experience design is *n*, and the random position of sports equipment is *L*=(*x*_*i*_), *x*_*i*_, *y*_*i*_ represents the relationship between experience design and sports equipment and *z*_*i*_ represents the influencing factors, then the initial position of sports equipment is as

(4) $$\begin{array}{c} L_{i}\left(x_{i}\right)=w\cdot K\left(x_{i}\right)+\text{rand}\left(0,1\right)K\left(x_{\text{jmax}}\right), \end{array}$$

where *x*_*i*_, *y*_*i*_, and*z*_*i*_ of any position *x*_*j*max_ are the maximum values of influencing factors and rand(0,1) is random numbers in the range of [0,1].

The ergonomic analysis indicators of sports equipment are randomly selected, and cross-design is carried out, so as to update the overall data of sports equipment. Under the constraint of satisfaction degree, the greedy strategy is used to obtain the optimal experience design that accords with the weight. The calculation process is given as

(5) $$\begin{array}{c} \Delta L_{i}\left(x_{i}\right)=\frac{w\cdot K\left(x_{i}\right)+\varphi_{ijz}\left(\Delta x_{io}\right)}{\sum \lambda \cdot \leq K\left(x_{i}|\right)}, \end{array}$$

where *o* ∈ [0, *n*/2], *i* ∈ [0, *n*], *φ*_*ijz*_ ∈ (−1,1), and *k* ≠ *i*.

The function of sports equipment is to select the best sports equipment by probability *p*_*i*_ and cycle strategy, and design the neighborhood around the better sports equipment to obtain the optimal experience design that meets the threshold [9]. The calculation process is

(6) $$\begin{array}{c} \left\{\begin{array}{c} p_{i}=\frac{K\left(x_{i}\right)}{\sum_{i,j,k}^{n}\left[K\left(\Delta x\right)|\gamma \right]},\\ K\left(\cdot \right)=\frac{1}{F\left(\cdot \right)}\;F\left(\cdot \right)\geq 0,\\ K\left(\cdot \right)=1+s.t.\left(\cdot \right)\;F\left(\cdot \right)<0. \end{array}\right. \end{array}$$

Among them, it is a moderate function of different influencing factors.

If the sports equipment design has not obtained the optimal experience design after infinite cycle adjustment, that is, the experience design matrix is 0, the sports equipment experience design will be abandoned, and the sports equipment function will be changed into the material analysis of sports equipment [10], and the new sports equipment materials, safety, and price will be randomly analyzed according to formula (4) for the next design.

(7) $$\begin{array}{c} \rho =\min\sum \Delta \nu_{i}\cdot e, \end{array}$$

where Δ*ν*_*i*_ is the inertia value of *i* position updates.

The dynamic adjustment of experience design optimization degree. In the initial stage, the materials of sports equipment cannot guarantee the overall design, which may fall into local design “trap” and reduce the overall performance of the algorithm [11]. Therefore, in the process of adjusting the experience design of sports equipment, we should try our best to expand the design scope, narrow the design scope near the optimal experience design, and constantly adjust the range. Some scholars adjust the optimization degree *ρ* of experience design linearly to reduce the randomness of the amplitude, but it falls into design error near the optimal experience design. In order to make up for the deficiency of experience design adjustment mentioned above, this article introduces dynamic adjustment factor*ν*, and its calculation formula is given as

Ergonomic analysis and the renewal of sports equipment functions can be changed into the following formula:

(8) $$\begin{array}{c} \Delta L\left(x_{i}\right)=w\cdot K\left(x_{i}\right)+\nu_{ijz}K\left(\Delta x_{ik}\right). \end{array}$$

From formula (7), *F*(*x*_*i*_, *y*_*i*_, *z*_*i*_)/∑*F*(*x*_*i*_, *y*_*i*_, *z*_*i*_) can be seen that the value is relatively small and the value *ν* is relatively large in the initial stage, which can expand the design range of ergonomic analysis [12] and keep the diversity of experience design adjustment. In the later stage of design, *ν* is relatively small, which narrows the design scope, improves the neighborhood design ability of ergonomic analysis, and enhances the dynamic design performance of the algorithm.

It can be seen from Figure 1 that the dynamic adjustment of experience design amplitude can accurately determine the global extreme value, and the extreme value is in the best effect of experience design sample experience design in the logistics chaos theory. Therefore, the dynamic adjustment of experience design optimization degree can make the data meet the requirements and improve the accuracy of calculation results.

The introduction of sports equipment factor. When the data of a certain sports equipment are collected many times and reach the mining limit, ergonomic analysis will be transformed into the material analysis of sports equipment, and a new experience design will be calculated [13]. Because of its strong randomness and poor resistance to uncertain factors, the bee colony algorithm will have errors in the early stage of experience design adjustment. The probability of bee colony error is positively correlated with the complexity of sports equipment. In order to make up for the above shortcomings, this article introduces sports equipment factor, reduces the complexity of sports equipment through probability density function, and helps bees to reduce early design errors. The calculation formula of the function is given as

(9) $$\begin{array}{c} L\left(x_{i}\right)=\frac{F\left(x_{i}\right)/\sum F\left(x_{i}\right)}{\pi {\sum_{i,k=1}^{+\infty }\left|K\left(\Delta x_{\text{ik}}\right)\right|}^{2}}. \end{array}$$

When *F*(*x*_*i*_, *y*_*i*_, *z*_*i*_)/∑*F*(*x*_*i*_, *y*_*i*_, *z*_*i*_) is 1, *F*(*x*_*i*_) is the standard distribution function of sports equipment Cauthy (0,1). At that time, the design complexity of sports equipment experience was the highest; otherwise, the complexity was the lowest [14]. Because Cauthy (0,1) tends to extremum at a slower speed than Gauss (0,1), it can effectively reduce the occurrence rate of early local extremum. Moreover, the peak value of Cauthy (0,1) is smaller than that of Gauss (0,1), which can improve the resistance of the function to uncertain factors. Based on the above analysis, the sports equipment experience design formula can be expressed as follows:

(10) $$\begin{array}{c} \Delta L_{i}=K\left(x_{i}\right)+\text{Cauthy}\left(0,1\right)K\left(\Delta x_{ik}\right). \end{array}$$

### 2.3. Dynamic Adjustment Strategy Analysis

Improved version of dynamic adjustment strategy. The reasonable choice of dynamic adjustment strategy is the main index of experience design. Ergonomic analysis, dynamic adjustment among sports equipment functions, sports equipment materials, safety, price, appearance, and other indicators can not only balance the relationship between global design and local design, but also improve the corresponding design ability [15]. From formula (8), we can see that in the initial design of sports equipment, we pay great attention to the global design ability, and in the later design, we pay attention to the local design, so different bees should dynamically choose the experience design according to the conditions.

(1) Ergonomic experience design is given as
  (11) $$\begin{array}{c} \Delta L_{i}\left(x_{i},y_{i},z_{i}\right)=\sum_{t}\Delta L_{i-1}\left(x_{i-1}\right)+\text{Cauthy}\left(0,1\right). \end{array}$$
(2) Experience design of equipment function is given as
  (12) $$\begin{array}{c} \Delta L_{i}\left(x_{i}\right)=\sum_{t}\Delta L_{i-1}\left(x_{i-1}\right)+\text{Cauthy}\left(0,1\right). \end{array}$$
(3) Experience design of equipment safety is given as
  (13) $$\begin{array}{c} \Delta L_{i}\left(x_{i}\right)=\sum_{i=1,t}^{n/2}\Delta L_{i-1}\left(x_{i-1}\right)+\text{Cauthy}\left(0,1\right). \end{array}$$
(4) Experience design of equipment price is given as
  (14) $$\begin{array}{c} \Delta L_{i}\left(x_{i}\right)=\sum_{t}\Delta L_{i-1}\left(x\right)\cdot F\left(x\right)+\text{Cauthy}\left(0,1\right)K\left(\Delta x_{i-1k}\right). \end{array}$$
(5) Experience design of equipment appearance is given as
  (15) $$\begin{array}{c} \Delta L_{i}\left(x_{i}\right)=\frac{\sum_{t}\Delta L_{i-1}\left(x\right)}{F\left(y\right)+\text{Cauthy}\left(0,1\right)K\left(\Delta x_{i-1k}\right)}. \end{array}$$
(6) Experience design of equipment and materials is given as
  (16) $$\begin{array}{c} \Delta L_{i}\left(x_{i}\right)=\sum_{t}\Delta L_{i-1}\left(x\right)+\text{Cauthy}\left(0,1\right)K\left(\Delta x_{i-1k}\right), \end{array}$$

where *t* is the adjustment time of bee colony.

In this article, the artificial bee colony algorithm is improved in two aspects: on the one hand, every time the sports equipment changes, under the constraints of weight designed *w* for experience and threshold designed *λ* for experience [16], the bee colony randomly selects strategies from five models and completes multiple collection of sports equipment. In the later stage of sports equipment design, the design space is gradually reduced, and the neighborhood design is carried out, and the diversity of bees is maintained to improve the global design ability. On the other hand, it balances the global and local design capabilities of the bee colony and incorporates the updated inertia value Δ*ν*_*i*_, moderation function *F*(*x*_*i*_), and Lagrangian multiplier function to design the best sports equipment more quickly.

Colony coordination is the main way to realize dynamic adjustment. Based on the dynamic adjustment of colony, this algorithm constructs a dynamic distributed coordination strategy [17]. Different subpopulations employ different dynamic cooperation strategies, complex parameters, and manipulations. The bee colony is randomly divided into five subgroups, and each subgroup represents a subspace. In each iterative process, subgroups will randomly choose different collaborative schemes. After each sports equipment is collected, compare the satisfaction value of different subgroups and the complexity of sports equipment, and record the global optimal position; other sub-bees gather towards the optimal experience design to improve the design efficiency of the best sports equipment.

### 2.4. Fusion of Logistic Chaos Theory and Artificial Bee Colony Algorithm

Because of the wide range of applications of the bee colony theory, we should adopt corresponding search strategies for different problems. The improved bee colony algorithm proposed in this article is based on the design experience of ice and snow sports equipment [18], so it is necessary to put forward corresponding constraints on the bee colony algorithm, namely, threshold and weight, to ensure the accuracy of the final calculation results meets the requirements. The implementation steps of this algorithm are shown in Figure 2.

  Step 1: determine the structure and complexity of sports equipment. According to the characteristics of practical problems, the nonlinear distribution structure of sports equipment is determined.
  Step 2: get the data of ice and snow sports equipment. According to the relevant parameters, the data of ice and snow sports equipment are obtained. The number of sports equipment and bee colony are same, which are n = 40 Δ*ν*_*i*_ ∈ [0.2, 0.9], and Cauthy(0,1) ∈ [0.11, 0.53] the iteration times *m* is 40.
  Step 3: determine the satisfaction function. The artificial bee colony is generated randomly by using the chaos theory of logistics, and its experience is designed into the influencing factor space, and the initial experience design weight *w* and experience design threshold *λ* are obtained. According to the application experience design of complex ice and snow sports equipment, *w* = 0.22 and *λ* = 0.92. Through formulas (3) ∼ (7), the artificial bee colony is improved, and the satisfaction value of each sports equipment is calculated.
  Step 4: calculate the global and local optimal experience design. The satisfaction degree is obtained, and the optimal global position is compared with the local optimal experience design of each subpopulation.
  Step 5: iterate of sports equipment and material update of sports equipment.The factors of sports equipment need to be dynamically adjusted and analyzed. The analysis method is to randomly select one of the five adjustment schemes for analysis. The integration of sports bad evaluation factor is C and inertia weight is Δ*ν*_*i*_ by formula (2) and formula (7).
  Step 6 (dynamic cooperative adjustment of each subpopulation): after a sports equipment experience, select the best global position, share the experience design with other sub-bees, analyze the best experience design, and adjust the neighborhood experience design.
  Step 7: judge whether the sports equipment reaches the maximum value *m* and whether the iteration times reach *m*. If it has been reached, repeat steps 1 to 5; otherwise, stop the adjustment of experience design, and return to threshold, weight, and global optimal experience design.

## 3. Empirical Analysis

### 3.1. Model Performance Analysis

In order to further verify the performance of the improved bee colony model, four benchmark analysis functions are selected, which are ergonomics, equipment function, safety, price, and appearance. The analysis process is as follows.

(1) Ergonomic function is given as
  (17) $$\begin{array}{c} f\left(x\right)=\sum_{i=1}\frac{x_{i}{}^{2}}{10}+1. \end{array}$$
(2) Equipment function is given as
  (18) $$\begin{array}{c} f\left(x\right)=\sum_{i=1}x_{i}{}^{2}+\kappa . \end{array}$$
(3) Security function is given as
  (19) $$\begin{array}{c} f\left(x\right)={\text{e}}^{\left(1/n\right)\sum_{i=1}\cos\left(2\pi x_{i}\right)}. \end{array}$$
(4) Price and appearance function is given as
  (20) $$\begin{array}{c} f\left(x\right)=1+\sum_{i=1}\frac{x_{i}{}^{2}}{4000}, \end{array}$$

where |*x*_*i*_| ∈ [0,600], *i* is 1, 2. Get the minimum value 0 at (0, 0). In this article, the parameters of the simulation experiment are set: the total number of sports equipment is 100, the iteration times are 100, the mining limit is 20 times, the maximum update inertia value Δ*ν*_max_=1.2, and the minimum inertia valueΔ*ν*_min_=0.2, and the result is the average of 100 iterations. The operation results of the four analysis functions are shown in Table 2.

It can be seen from Table 1 that the improved bee colony model is superior to the artificial bee colony algorithm, and its global optimal value is closer to the theoretical optimal value. Moreover, the value range, average value, and calculation error of the improved bee colony model are smaller than those of the artificial bee colony algorithm. In order to more intuitively reflect the experience design adjustment performance of the analysis function in 4, the following convergence graph is given, as shown in Figures 3∼6.

As can be seen from Figures 3∼6, the experience design of the improved bee colony model has faster adjustment speed and better stability, which is superior to the artificial bee colony algorithm. Therefore, the improved bee colony model has better performance in calculation speed and accuracy, and the calculation process is more stable.

### 3.2. Sample Data Processing

In this article, ice and snow sports equipment is selected as the research experience design sample. The sports time is from January 20, 2022, to May 10, 2022, and the collection interval is 4 hours. After preliminary data collation, 45 rows of data and 12 types of ice and snow sports equipment were obtained. According to the experience standard, the application experience design of ice and snow sports equipment is judged, and the ice and snow sports equipment is divided into four categories: ergonomics, equipment function, equipment safety, and equipment price. According to the theory of bee colony, combined with the application data of ice and snow sports equipment, the accuracy of the model proposed in this article is verified. To avoid redundancy in collecting data, call the function to replace duplicate data and keep the complexity of collecting data. The results are shown in Table 3.

The first 1/2 of the total number of experience design samples is taken as the training experience design samples, and the last n/2 is taken as the test set for experimental comparison.

### 3.3. Experimental Results

According to the experimental situation, the data complexity distribution of ice and snow sports equipment is determined, the maximum iteration times are *M* = 40, and other parameters are set the same. This article presents the classification results of the model for the application experience design of complex ice and snow sports equipment, as shown in Figure 7.

Through comparative analysis, we can see that the classification of experience design samples of the improved bee colony model is discrete, which is closer to the actual application experience design distribution of ice and snow sports equipment, while the classification of experience design samples of the artificial bee colony algorithm is relatively concentrated, which cannot meet the needs of actual classification. In addition, the sample distribution of experience design of improved bee colony model is not affected by complexity, while the sample distribution of experience design of the artificial bee colony algorithm is obviously affected by complexity and becomes more concentrated with the increase of complexity. The reason is that the improved bee colony model increases the complexity processing coefficient and integrates uncertain factors Cauthy(0,1) into the experience design. At the same time, the satisfaction function is used to adjust the experience design.

In order to further prove the effectiveness of the model proposed in this paper, other comparative models are introduced for comparative analysis: (1) artificial bee colony algorithm, (2) logistic chaos theory combined with the artificial bee colony algorithm, and (3) logistic chaos theory combined with logistic chaos theory. This paper improves the bee colony model, and the results are shown in Figure 8.

It can be seen from the above figure that the satisfaction value of the improved bee colony model is the highest and reaches the limit at the earliest. Under the same complexity, the improved bee colony model has higher stability, followed by the artificial bee colony algorithm, logistic chaos theory combined with the logistic chaos theory, and logistic chaos theory combined with the artificial bee colony algorithm. The reason is that the logistic chaos theory reduces the influence of complexity on calculation results, and the logistic chaos theory provides different adjustment strategies to improve the accuracy of judgment results of ice and snow sports equipment, which is consistent with relevant research Fan and Ding [19]. The turning point of the improved bee colony algorithm appears in 50 iterations, and the turning point appears once. Compared with the improved bee colony, the turning point of the artificial bee colony algorithm appears 45 iterations and 80 iterations, and the turning point appears twice. The change range of the improved bee colony algorithm is 3% and that of the artificial bee colony algorithm is 5%, which further shows that the improved risk algorithm is superior to the artificial bee colony algorithm. The reason is that the improved bee colony algorithm preprocesses the dataset of sports equipment application experience design and combines the chaos theory to simplify the data and reduce the interference of redundant data. From the application experience of complex ice and snow sports equipment design ice and snow sports equipment types, the accuracy of different algorithms is analyzed, and the results are shown in Table 4.

As can be seen from the above table, the judgment rate of ice and snow sports equipment of the improved bee colony model is higher, and the accuracy rate does not change with the change of ice and snow sports equipment types. The main reason is that the dynamic analysis of sports equipment factor on experience design samples makes its continuous calculation time shorter and can change the types of ice and snow sports equipment more flexibly. Therefore, dynamic sports equipment can not only reduce the impact of complexity on the results, but also quickly realize the accurate analysis of different types of ice and snow sports equipment.

## 4. Concluding Remarks

There are many experiences in the application design of ice and snow sports equipment, and a single statistical method cannot be accurately analyzed. In order to better carry out the corresponding research Cheng [20], this article combines the chaos theory model with the bee colony algorithm and comprehensively judges the experience design results through bionic algorithm. In the research process, corresponding constraints are added to the threshold and weight settings of the bee colony algorithm to ensure the accuracy of the calculation results [21]. In addition, by preprocessing the previous data and eliminating irrelevant data content, the speed of calculation can be improved. In the actual analysis process, it is found that the improved bee colony algorithm is superior to the artificial bee colony algorithm in calculation accuracy, data variation range, data convergence speed, and analysis index accuracy. Moreover, MATLAB simulation results show that the stability and convergence of the improved bee colony algorithm are more than 95%, which is better than 90% of the artificial bee colony algorithm. Therefore, the improved bee colony algorithm can adapt to different complexity and types of ice and snow sports equipment and has high global design ability.

## Figures and Tables

**Figure 1:** Dynamic adjustment result of design amplitude.

**Figure 2:** Implementation flow of improving the bee colony model.

**Figure 3:** Convergence curve of the experience design adjustment of ergonomic analysis function.

**Figure 4:** Convergence curve of the experience design adjustment of equipment function analysis function.

**Figure 5:** Experience design adjustment convergence curve of security analysis function.

**Figure 6:** Convergence curve of experience design adjustment of price and appearance analysis function.

**Figure 7:** Classification results of application experience design samples of ice and snow sports equipment.

**Figure 8:** Comparison of satisfaction values of different methods. *Note*. The red line is the improved bee colony algorithm proposed in this paper, and the blue line is the standard artificial bee colony algorithm.

**Table 1:** Investigation results of the application experience design of ice and snow sports equipment in 2022.

Material item	Experience design complexity	Experience requirements
Sleigh	0.23	Hight
Sledge	0.27	Media
Snowboard	0.32	Media
Goggles	0.41	Media
Helmet	0.13	Hight
Snowshoe	0.23	Media
Snow tire	0.31	Media
Snow suit	0.42	Media
Veneer	0.21	Hight
Ice hockey	0.54	Hight
Curling	0.23	Hight
Holistic	0.62	Hight
Veneer	0.23	Hight
Ice hockey	0.51	Hight
Curling	0.21	Hight
Holistic	0.32	Hight

Data Source: Questionnaire Survey, Interview Questionnaire

**Table 2:** Results of different analysis functions.

Function	Method	Ergonomics	Equipment function	Security	Price	Appearance	Best experience design
Ergonomics	Artificial bee colony algorithm	1.51	1.34	1.42	0.73	0.64	0
	Improved bee colony model	0.41	0.24	0.32	0.38	0.28	0

Equipment function	Artificial bee colony algorithm	1.68	1.42	1.42	0.36	1.43	2
	Improved bee colony model	0.51	0.32	0.45	0.16	0.28	0

Security	Artificial bee colony algorithm	1.8499E-05	1.3454E-05	1.42	1.58	1.27	0
	Improved bee colony model	0.6818E-05	0.3124E-05	0.51	0.53	0.23	2

Price and appearance	Artificial bee colony algorithm	1.6818E-05	1.5136E-05	1.59	1.51	1.28	0
	Improved bee colony model	0.5236E-05	0.1295E-05	0.21	0.21	0.31	2

**Table 3:** Data types and proportion of ice and snow sports equipment collected.

Clustering of ice and snow sports equipment	Amount of data	Proportion (%)
Ergonomics (2)	43	22.05
Instrument function (2)	32	15.90
Instrument safety (3)	23	11.79
Instrument price (3)	38	11.26
Color appearance of instrument (2)	22	23.3

**Table 4:** Judgment accuracy of different ice and snow sports equipment types.

Clustering of ice and snow sports equipment	Improved bee colony model		Artificial bee colony algorithm	
	Accuracy	Time	Accuracy	Time
Ergonomics	99.94	98.93	97.92	96.91
Instrument function	99.97	98.92	98.97	98.90
Instrument safety	99.91	95.94	95.93	92.91
Instrument price	99.94	97.92	94.93	95.96

## Data Availability

The data used to support the findings of this study are available from the corresponding author upon request.

## References

[1] Kher G., Swami A., Ahlawat N., Kumar S., Yadav A. S. (2022). Inventory model for decay items with safe chemical storage and inflation using artificial bee colony algorithm. *International Journal of Applied Management Science*.

[2] Unzeitig G., Eggmann F., Filippi A. (2022). Dental and general injuries among ski and snowboard instructors in Switzerland, Germany, and Austria-A questionnaire-based study. *Clinical and Experimental Dental Research*.

[3] Stuart C. A., Brubacher J. R., Yau L., Yip R., Cripton P. A. (2020). Skiing and snowboarding head injury: a retrospective centre-based study and implications for helmet test standards. *Clinical Biomechanics*.

[4] Srinivas S., McLoughlin R. J., Hazeltine M. D. (2021). Pediatric snow sport injuries differ by age. *Journal of Pediatric Surgery*.

[5] Signetti S., Nicotra M., Colonna M., Pugno N. M. (2019). Modeling and simulation of the impact behavior of soft polymeric-foam-based back protectors for winter sports. *Journal of Science and Medicine in Sport*.

[6] Sekman D., Karakaya V. (2022). Controlling chaos for multistep iteration process and its special iterations in discrete dynamical systems. *International Journal of Bifurcation and Chaos*.

[7] Schmolke A., Abi-Akar F., Perkins D., Galic N., Hinarejos S. (2019). Addressing multiple factors impacting honey bee colonies in large colony feeding studies with a mechanistic honey bee colony model. *Abstracts of Papers American Chemical Society*.

[8] Requier F., Rome Q., Chiron G. (2019). Predation of the invasive Asian hornet affects foraging activity and survival probability of honey bees in Western Europe. *Journal of Pest Science*.

[9] Nicotra M., Moncalero M., Messori M., Fabbri E., Fiorini M., Colonna M. (2014). Thermo-mechanical and impact properties of polymeric foams used for snow sports protective equipment. *Procedia Engineering*.

[10] Nardo L. G., Nepomuceno E. G., Bastos G. T., Santos T. A., Butusov D. N., Arias-Garcia J. (2021). A reliable chaos-based cryptography using Galois field. *Chaos*.

[11] Minucci J. M., Curry R., DeGrandi-Hoffman G., Douglass C., Garber K., Purucker S. T. (2021). Inferring pesticide toxicity to honey bees from a field-based feeding study using a colony model and Bayesian inference. *Ecological Applications: A Publication of the Ecological Society of America*.

[12] Magal P., Webb G. F., Wu Y. X. (2020). A spatial model of honey bee colony collapse due to pesticide contamination of foraging bees. *Journal of Mathematical Biology*.

[13] Liu Z. L. (2022). Research on the possibility of smart wearable devices in ice and snow sports based on wireless network. *Wireless Communications and Mobile Computing*.

[14] Korzeniewski K., Pokorna-Kalwak D. (2020). Extreme travel medicine. *Family Medicine & Primary Care Review*.

[15] Jan A. M., Parah S. A., Malik B. A. (2022). IEFHAC: image encryption framework based on hessenberg transform and chaotic theory for smart health. *Multimedia Tools and Applications*.

[16] Hume P. A., Lorimer A. V., Griffiths P. C., Carlson I., Lamont M. (2015). Recreational snow-sports injury risk factors and countermeasures: a meta-analysis review and haddon matrix evaluation. *Sports Medicine*.

[17] Hachana O., El-Fergany A. A. (2022). Efficient PEM fuel cells parameters identification using hybrid artificial bee colony differential evolution optimizer. *Energy*.

[18] Fraccaroli L., Concli F. (2020). Introduction of open-source engineering tools for the structural modeling of a multilayer mountaineering ski under operation. *Applied Sciences*.

[19] Fan C. L., Ding Q. (2021). Analyzing the period distribution of digital chaos with graph theory. *Physica Scripta*.

[20] Cheng L. (2022). Implementation of snow and ice sports health and sports information collection system based on internet of things. *Journal of Healthcare Engineering*.

[21] Chen N. Y., Yang Y. P., Jiang Y. F., Ao Y. F. (2020). Injury patterns in a large-scale ski resort in the host city of 2022 Winter Olympic Games: a retrospective cross-sectional study. *BMJ Open*.

